The article "Research on Citizen Participation in Government Ecological Environment Governance Based on the Research Perspective of “Dual Carbon Target”" was published in 2022. Journal: J Environ Public Health.

# Research on Citizen Participation in Government Ecological Environment Governance Based on the Research Perspective of “Dual Carbon Target”

**DOI:** 10.1155/2022/5062620

**Published:** 2022-06-20

**Authors:** Shiyong Chen, Nan Liu

**Affiliations:** ^1^School of Marxism, Southwest Medical University, Luzhou 646000, Sichuan, China; ^2^School of Law, Southwest Medical University, Luzhou 646000, Sichuan, China

## Abstract

As the people's demand for a better life is getting higher and higher, citizens' requirements for the rural ecological environment are also constantly improving. At present, the deterioration of many rural environments and the cross-flow of sewage have brought great challenges to the governance of the rural ecological environment. Therefore, the improvement in the ability and level of rural ecological environment governance is the key to winning the battle of rural ecological environment governance, and the participation of citizens in rural ecological environment governance is even more crucial to the improvement in the ability and level of rural ecological environment governance. At present, academic achievements on rural ecological environment governance are increasingly enriched, but there are few academic achievements on rural ecological environment governance from the perspective of citizen participation. Since public participation in ecological environment governance is still in the initial stage of development, there are many factors that affect the effective implementation and development of public participation in the ecological environment. For example, various factors such as the imperfect legal system related to citizens' participation in rural ecological environment governance, weak awareness of citizen participation, and difficulty in determining the methods of citizen participation seriously hinder citizens' participation. Improve the theme awareness and ability of citizens to participate in ecological environment governance and to improve the citizen participation mechanism in my country's rural ecological environment governance. By analyzing and discussing the problems and countermeasures of public participation in environmental governance in my country, it is of positive significance to promote citizens' participation in ecological environmental governance.

## 1. Introduction

The year 2020 marks the 15th anniversary of General Secretary Xi Jinping's statement that “clear waters and lush mountains are invaluable assets” and is also a decisive year in China's battle against pollution. Highlighting the key points of ecological and environmental governance and making up the weak points of ecological and environmental governance are the key points in the battle against pollution. China's rural areas are not only populous, but also wide and diverse, which is not conducive to the rapid improvement in rural ecological environment governance level. In 2021, the seventh national census showed that the population living in rural areas was 509.79 million, accounting for 36.11%. The huge population has become one of the great obstacles to improving the level of rural ecological environment management in China.

The article "Research on Citizen Participation in Government Ecological Environment Governance Based on the Research Perspective of “Dual Carbon Target”" was published in 2022. Journal: J Environ Public Health.

After citizens' participation in rural ecological environment governance, the role of citizens has undergone a fundamental change: citizens have changed from the role of “being controlled” to the role of “being in charge of their own affairs” and “self-examination and introspection.” Therefore, allowing citizens to participate in the governance of the local ecological environment is not only the transformation of citizens as “masters of their own affairs,” but also the self-satisfaction of citizens for political rights, enabling them to experience the rights and responsibilities granted by the constitution. Citizens are the destroyers and guardians of the local ecological environment [1]. Only by changing citizens' way of life and production, enhancing citizens' awareness of environmental protection, enabling citizens to understand the ways and means of protecting and managing the ecological environment, and changing their inherent way of life, can citizens become real “green citizens.” By allowing citizens to participate in rural ecological environmental governance, we can further cultivate the backbone of China's environmental protection. Standardizing the ways and methods of participation of all parties can not only promote the development of rural ecological environmental governance and save social governance costs, but also achieve a virtuo [2].

## 2. Concept Definition and Theoretical Basis

### 2.1. Concept Definition

#### 2.1.1. Ecological Governance

Ecological governance is the process of rectifying, cleaning up, restoring, and beautifying the ecological environment in the process of ecological civilization construction, with the goal of achieving ecological civilization; green technology innovation as the driving force; and government-led social organizations, enterprises, and institutions; and individual citizens, the process of participation [3]. Through ecological environment governance, behaviors that affect or even cause serious damage to the ecological environment should be deeply managed and constructed under the condition of maintaining a stable ecological environment. To a certain extent, improving the ecological environment can comprehensively improve the living environment of citizens.

The article "Research on Citizen Participation in Government Ecological Environment Governance Based on the Research Perspective of “Dual Carbon Target”" was published in 2022. Journal: J Environ Public Health.

#### 2.1.2. Citizen Participation

The domestic definitions of civic participation mainly include: that public participation in all activities that citizens try to influence public policy and civic life; and that civic participation refers to a series of behaviors related to citizens trying to influence government decision-making activities through channels within the political system. Public participation emphasizes the two-way communication and consultative dialogue between decision makers and stakeholders affected by the decision [4]. Based on the above definition, civic participation has the following characteristics: citizens participate through certain participation mechanisms or channels, citizens influence policy systems and public affairs or affect civic life, and citizen participation is a positive behavioral activity. Therefore, this article defines citizen participation in ecological governance as a series of positive behaviors in which citizens affect policy systems, public affairs, or citizens' lives through certain participation mechanisms or channels.

#### 2.1.3. Dual Carbon Goals

The “dual carbon” target is my country's updated nationally determined contribution strengthening target in accordance with the “Paris Agreement” and a long-term low greenhouse gas emission development strategy for the mid-21^st^ century. It climbs from fast to slow, fluctuates at an inflection point of zero annual growth, and then continues to decline until anthropocentric sources and sinks balance out. The process from carbon peaking to carbon neutrality is the process of carbon dioxide emissions from relative decoupling to absolute decoupling of economic growth. My country strives to achieve the peak of carbon dioxide emissions before 2030, the carbon dioxide emissions per unit of GDP will drop by more than 65% compared with 2005, the proportion of nonfossil energy in primary energy consumption will reach about 25%, and the total installed capacity of wind power and solar power will reach more than 1.2 billion kilowatts and achieve carbon neutrality by 2060. During the “14^th^ Five-Year Plan” period, energy consumption and carbon dioxide emissions per unit of GDP will be reduced by 13.5% and 18%, respectively. Promoting the decarbonization, electrification, and intelligence of the energy and power system; the conversion of low-carbon fuels (in areas that cannot be electrified); and the application of negative emission technologies are the basic paths to achieve carbon neutrality before 2060.

In recent years, my country is seeking a more sustainable, inclusive, and resilient economic growth mode and already has the objective conditions to achieve the peak of carbon emissions before 2030. As the only major economy to achieve positive economic growth in 2020, my country shoulders the heavy responsibility of leading the “green recovery” of the world economy. In 2020, my country's total economic output will account for about 17.39% of the world's total, and carbon dioxide emissions will account for about 29% of the world's total emissions. In 2020, my country's total economic volume has reached a major step of one trillion yuan, and the strong national comprehensive strength has laid a solid economic foundation for the realization of the “dual carbon” goal. Achieving carbon peaking and carbon neutrality is an extensive and profound economic and social transformation, and the Party Central Committee has a clear understanding of this big test. Compared with developed countries, my country has a tighter time frame, greater scope, more difficulties, and extremely arduous tasks to achieve the “dual carbon” goal. It requires both courage to face adjustment and wisdom to overcome difficulties. There is a long way to go to create a new paradigm of development.

The article "Research on Citizen Participation in Government Ecological Environment Governance Based on the Research Perspective of “Dual Carbon Target”" was published in 2022. Journal: J Environ Public Health.

### 2.2. Theoretical Basis

#### 2.2.1. Synergy Theory

Synergy theory mainly studies how an open system that is far from the equilibrium state spontaneously emerges an ordered structure in time, space, and function through its own internal synergy when there is material or energy exchange with the outside world. Synergy theory is based on the latest achievements of modern science—system theory, information theory, cybernetics, and catastrophe theory—absorbs a lot of nutrition from the theory of structural dissipation, and adopts the method of combining statistics and dynamics. Based on the analysis, a multidimensional phase space theory is proposed, a set of mathematical models and processing schemes are established, and the common law of the transition from disorder to order in various systems and phenomena is described in the transition from micro to macro. Mainly biased towards three aspects, namely, conflicting multiple and contradictory subjects; transforming contradictions into cooperation methods; and achieving a harmonious, collaborative, and win-win situation, the three complement each other and are indispensable. Therefore, the author believes that in citizens' participation in the governance of the rural ecological environment, in order to adjust the conflicts of interests caused by the ecological environment problems of multiple subjects such as “citizens, township grassroots governments, rural production and operation cooperatives (capital), and nongovernmental environmental protection organizations,” a mutual benefit must be achieved. Multiple measures and multiple ways should be coordinated with rural ecological environment governance issues to achieve a win-win situation and a beautiful ecological environment. Citizens' participation in rural ecological environment governance from the perspective of synergy is in essence; under the condition of consensus and coordination of multiple subjects, grassroots governments improve and decentralize power, grassroots people coordinately manage ecological and environmental affairs and improve the collaborative management under the grassroots mass power system. The synergy theory has come to fruition in my country and is playing an important role in all aspects of social governance.

The article "Research on Citizen Participation in Government Ecological Environment Governance Based on the Research Perspective of “Dual Carbon Target”" was published in 2022. Journal: J Environ Public Health.

#### 2.2.2. Governance Theory

American Scholar Box is a pioneer of civil governance theory. In his book “Civil Governance: Leading American Communities in the 21^st^ Century,” he criticized some views of the new public management theory and repositioned citizens, government decision makers, and administrative professional management. The role of three persons are as follows: citizens become direct participants and controllers of public affairs because of their positive citizenship, not just service objects of government affairs; government decision makers are transformed from single commanders and controllers to active promoters; and administrative professional managers should not try to control the government and public institutions, but should play a supporting role in promoting citizen participation. At the same time, it is believed that the government should transform the bureaucracy in the traditional sense, empower citizens with more rights, and put forward four principles of citizen participation, namely scale, democracy, rationality, and responsibility. Citizens can only be guided by these four principles. Public participation will play its effectiveness [5].

Governance theory strongly advocates diversified management: usually, the cooperation between the government, social organizations and groups, the market, and individual citizens is strengthened by means of divisions such as levels and stages to form multiple co-governance subjects. In addition, through the emphasis on government reform and function transformation, and the introduction of competition mechanism advocacy, various governance bodies are interconnected and independent of each other and share responsibilities to achieve common goals [6]. The proposal of governance theory is a manifestation of the progress of human thought, and it has been applied in various fields around the world, namely social governance, population governance, environmental governance, ecological governance, and network governance. Therefore, pluralistic co-governance is a new paradigm of ecological governance, and it is also a process of collective participation and collective decision-making. Citizen participation in ecological governance is a manifestation of the diversification of governance subjects. Therefore, based on governance theory, this article explores the issue of citizen participation in the ecological governance of Ziwuling National Forest Park in Gansu.

The article "Research on Citizen Participation in Government Ecological Environment Governance Based on the Research Perspective of “Dual Carbon Target”" was published in 2022. Journal: J Environ Public Health.

#### 2.2.3. Stakeholder Theory

Stakeholder theory was gradually developed in Western countries around the 1960s, and its influence expanded rapidly after the 1980s, began to influence the choice of corporate governance models in the United States and the United Kingdom, and promoted corporate governance, changes in management style. The reason for the emergence of the stakeholder theory is its profound theoretical and practical background. The key point of the stakeholder theory's foothold is that it believes that with the development of the times, the status of the owners of physical capital in the company is gradually weakening. The so-called weakening of the status of material owners means that stakeholder theory strongly challenges the traditional core concept that a company is owned by individuals and institutions that hold common stock in the company. Originally applied in the field of economic management, with the development of related research, this theory has gradually developed into the field of public management and has been widely used in the research of government, citizens, and nonprofit organizations in the third sector. In the environmental field, all citizens live in it. As the direct bearers of ecological changes, they have the most say in ecological governance in the face of ecological damage. Therefore, the stakeholder theory is an important theoretical basis for citizens to participate in ecological governance [7]. In order to realize the long-term development of the country in the government's ecological governance, it is necessary to incorporate multistakeholders into the ecological governance.

### 2.3. The Basic Status of Chinese Citizens' Participation in Rural Ecological Environment Governance

#### 2.3.1. Increasing Awareness of Environmental Protection

Comparing the “Citizens' Ecological and environmental Behavior Survey Report” for 2019 and 2020, the proportion of respondents to the topic of “concern about ecological environment” increased by 10%–20% (Figure 1).

It can be seen from the above picture that the ecological environment awareness of Chinese citizens is gradually improving, as shown in Figures 2 and 3. There are many channels for Chinese citizens to obtain information, among which the Internet, radio, and neighbors are important information sources. Specific information acquisition channels are shown in Figure 4. Although the respondents in the “Citizens' Ecological Environmental Behavior Survey Report” involved a large number of urban residents and township citizens, the 2019 “Report” clearly pointed out that the respondents were in different work units, indicating that urban and rural concerns. For differences in ecological environment information, compared with national or regional ecological environment information, citizens pay more attention to the ecological environment information that is closely related to their living places, as shown in Figures 5 and 6.

The article "Research on Citizen Participation in Government Ecological Environment Governance Based on the Research Perspective of “Dual Carbon Target”" was published in 2022. Journal: J Environ Public Health.

### 2.4. Enhanced Participation Ability

In recent years, the ability of Chinese citizens to participate in rural ecological environment governance has gradually increased, mainly reflected in the gradual enhancement of the public's behavior of “practicing” ecological environmental protection. The ability of Chinese citizens to practice ecological environment governance has risen. From the Survey Report on Citizens' Ecological Environment Behavior (2020), respondents generally believe that their environmental protection behavior is very important to protect the ecological environment. Therefore, citizens attach great importance to low-carbon travel and energy conservation and enthusiastically participate in supervision and reporting and environmental volunteering activities. However, the respondents' practice in the fields of green consumption, reducing pollution, paying attention to the ecological environment, and sorting garbage is relatively poor. However, compared with 2019, the practice of the public in my country has increased by about 10% as shown in Figure 7. The specific data are shown in Figure 8.

The rate of rural sewage treatment in China has increased. In 2019, according to relevant media reports, the sewage treatment rate in rural areas of Shanghai has reached 75%, and the phenomenon of sewage discharge in rural areas has been greatly improved, making it the highest sewage treatment rate in rural areas of China. China's garbage disposal capacity has increased. As shown in Figure 8, according to the data of the National Bureau of Statistics from 2012 to 2019, China's garbage harmless treatment capacity increased year by year. During the same period, the treatment capacity grew slowly and reached 240,128,000 tons in 2019, and its daily treatment capacity reached 869,875 tons.

### 2.5. Citizen Participation Channels Are Not Smooth

Citizens' participation in ecological governance has long been valued in Western countries, and the relevant laws and regulations are relatively complete. For example, the United States promulgated the “National Environmental Policy Law” as early as 1969, which guarantees citizens' right to participate in environmental protection. In addition, the developed countries, such as France and the United Kingdom, that have risen in the second industrial revolution have legally clarified the status of citizens' participation in environmental protection [7]. In these countries, citizens participate in ecological governance in various ways, and the participation channels are relatively smooth. They can participate through formal channels organized by government organizations, or through social organizations or spontaneous informal channels [8]. Participation methods provided by the government include hearings, seminars, and public surveys and timely release of relevant information on ecological governance; informal participation is led by social organizations and ordinary people, who participate in demonstrations, sign signatures, and contact the media; and the opinion is conveyed to government administrators. In contrast, the effective channels provided by local governments in my country are relatively simple; there are few channels for participating in environmental governance-related activities to truly play a role, and institutionalized channels such as symposiums and hearings are less open, especially in grassroots local governments, many of which are formalistic. At present, social environmental protection organizations have played an important role in ecological governance in Western countries. They have participated in ecological governance by raising funds, volunteering, and influencing government interest groups. However, in my country, social environmental protection organizations are far from developing. It is far behind developed countries, and its role is limited. Most of the grassroots people passively participate in government-led activities such as environmental protection popularization and publicity, but their active participation is poor, and the effectiveness of the participation path is not guaranteed. At present, the channels of participation of citizens in administrative decision-making in my country are not smooth, which leads to the prominent problem of disorder, the process of participation is more complicated, and the effect of participation is far from expected, which seriously affects the confidence and enthusiasm of citizens to participate in administrative decision-making. Due to the interference of various factors in real life, citizens' participation in administrative decision-making is seriously formalized, and the expected participation effect cannot be achieved.

The article "Research on Citizen Participation in Government Ecological Environment Governance Based on the Research Perspective of “Dual Carbon Target”" was published in 2022. Journal: J Environ Public Health.

On the one hand, poor participation leads to disorderly participation, which is mainly manifested in noninstitutionalized participation. Citizens who could have participated in administrative decision-making in a legal and standardized way, due to their own lack of understanding and biased thinking, forcibly participate in a disorderly manner to administrative decision-making. Among them, the most prominent ones are disorderly petitioning, illegal assembly, irrational participation through violence, and making rumors. Investigating the reason, we found that for citizens who participated in disorder, the deviation in ideology and understanding led to a certain misunderstanding of the government's open and reasonable behavior of allowing citizens to participate. Violent and malicious participation is an attempt to force the government to achieve its own goals through brutal means. These illegal, violent, and excessive behaviors will seriously damage social harmony and even endanger social security.

On the other hand, the lack of smooth participation channels has a negative impact on citizens' confidence in participating in administrative decision-making. Although citizen participation has been in-depth development in the process of building and developing a service-oriented government in recent years, in many cases, citizen participation is only a formality, and the rights and positive effects of citizen participation have not been fully exerted. In the Maoming PX incident, it was because of the lack of effective channels for participation, that the citizens finally took the method of protesting by marching. Although the development of the Internet has provided a convenient channel for citizens to participate, the effectiveness of local network participation at the grassroots level is still open to question, and the path for citizen participation is not smooth. Governance is also a long-term and arduous project. If this aspect cannot be effectively solved, it can be said that governance work is impossible [9]. There is still room for improvement in the willingness and participation of Chinese citizens, as given in Table 1.

### 2.6. Citizens Lack Ecological Knowledge

Ecosystem is a biological and environmental interrelated interaction and the formation of an organic and unified whole itself has certain cycle, if human needs are beyond the load of the ecosystem, will appear forests, grassland degradation, soil erosion, environmental pollution, climate anomalies, and species extinction phenomenon, affecting people's production and living. Human beings are an important factor in the cycle of the ecosystem, but for a long time, people have insufficient understanding of the ecological law and have not been alert to the ecological imbalance. They still blindly develop and utilize natural resources, causing the ecological environment in some areas to be difficult or impossible to recover and serious ecological problems [10]. Only when citizens have a scientific understanding of ecological knowledge, such as ecological environment, ecological system, ecological crisis and ecological law, can we better talk about the improvement in citizens' ecological awareness and the protection and governance of China's ecological environment [11]. My country is in the primary stage of socialism. By the end of 2020, a well-off society will be fully realized, which is also a critical period for the construction of a service-oriented government. There is still a big imbalance in the progress of social development, and there is also an imbalance in the overall quality of our citizens. The uneven comprehensive quality of citizens will be directly manifested as insufficient understanding of the content of policy issues, inability to make rational and correct judgments in choosing participation methods, and inability to fully understand the results of decision-making with a normal mentality. These phenomena will adversely affect the healthy development of civic participation and even damage the public interest. The comprehensive improvement in the comprehensive quality of citizens requires the joint efforts of society, the government, and individuals, and improving the comprehensive quality of citizens is an important prerequisite for improving the ability of citizens to participate and realizing democratic participation.

The article "Research on Citizen Participation in Government Ecological Environment Governance Based on the Research Perspective of “Dual Carbon Target”" was published in 2022. Journal: J Environ Public Health.

Ecological behavior is an actual behavior in which people put their understanding, cognition, and emotion of ecological environment in daily life into certain ecological practice. At present, Chinese citizens have a lot of bad environmental behaviors in their daily life. For example, the government advocates the concept of “low-carbon life,” but in real life, we see too many non-“low-carbon” behaviors of citizens: throwing away waste batteries, using disposable tableware, driving when going out, and being obsessed with fur [12]. In fact, low-carbon life involves people's clothing, food, housing, transportation, and other aspects; the long-formed living habits and consumption patterns cannot be the reason for citizens to reject low-carbon life, as long as they improve their living habits, take the initiative to restrain themselves, and save all kinds of resources around, they will leave everyone's “carbon footprint.” Otherwise, these nonenvironmental behaviors will become the root of ecological and environmental problems. Therefore, we should construct the daily ecological norms of citizens and develop good ecological behaviors of citizens.

The article "Research on Citizen Participation in Government Ecological Environment Governance Based on the Research Perspective of “Dual Carbon Target”" was published in 2022. Journal: J Environ Public Health.

### 2.7. Lack of Legal Guarantee for Citizen Participation

Gradually in recent years, the citizen participation in the form of diversity, in addition to being able to rely on the people's congress system, political consultative system and the grassroots autonomy system, and other countries outside the political system to participate in government administration, democratic appraisal government, government officials, online q&a, and policy hearing form also gradually rise, but in the construction of local government, a large part of become a mere formality, the lack of actual effect. In addition, citizen participation is usually related to policy development, water and electricity prices, and demolition of housing, but it is rare to apply it to ecological environment governance [13]. Some local governments believe that ecological governance is an activity with the government as the main executioner, and ordinary people have neither professional knowledge nor the ability to participate in it. Therefore, it is unnecessary to introduce the public into government governance. This led to the process of ecological management in local government, and there are no relevant laws and regulations to provide protection for citizen participation; the social reality of this lack of security makes some people to express their interests in the ecological regulation, of the unsoundness of informal ways involved in the government management, and also brought the government's governance. The deficiencies of the current legal system of citizen participation in China are mainly reflected in: (1) the constitutional guarantee of citizen participation is not perfect. The definition of citizen's participation right in the constitution of our country is vague and there is no guarantee provision, which is very unfavorable to the protection and development of citizen's participation right. Due to the lack of the right to guarantee the formal participation path, a large number of people have to participate in the informal path. Most participants do not get normative guidance, and the disorderly nature of informal participation leads to the formation of mass incidents and harm to public security. (2) The specific field of civic participation is not clear [14, 15]. Although the law guarantees citizens' participation, the current law does not specify the specific areas in which citizens can participate and does not specify what kind of government affairs the public can participate in, and if so, what procedures, processes, and channels should be used to participate, which are lacking in the current laws and regulations. To some extent, it hinders the actual participation of the public. (3) Lack of legal enforcement. The law points out the specific ways in which citizens can participate in State Administration in China, but it lacks legal effect in the specific implementation of participation. However, it is difficult to play a role in the actual process of government governance. Social forces and citizen groups can communicate with the state authorities through legal communication channels. Improving the legal system of citizen participation is an important prerequisite for the effective participation of citizens. Without the protection of the legal system, citizens' right to participate is easy to be ignored and trampled. The rule of law is a major national policy requirement of the country. In the process of social management, the government should further improve the citizen participation system and law according to the requirements of the times and the public. Let the public have the opportunity to participate in the government's actual ecological governance [16].

The article "Research on Citizen Participation in Government Ecological Environment Governance Based on the Research Perspective of “Dual Carbon Target”" was published in 2022. Journal: J Environ Public Health.

## 3. Suggestions on Strengthening Citizens' Participation in Ecological and Environmental Governance

### 3.1. Raising Citizens' Ecological Awareness

The experience of economic development and environmental protection in Western developed countries has given us a lot of enlightenment. To do a good job in cultivating citizens' ecological consciousness, we should broaden our international vision and draw lessons from foreign advanced ecological education experience. At the same time, we should combine China's specific national conditions and reality to find out the similarities between foreign countries and the cultivation of Chinese citizens' ecological consciousness and build a cultivation model with Chinese characteristics to shape the modern ecological consciousness of Chinese citizens, advocating the government-led training model. In 1970, more than 20 million people participated in the social demonstration of environmental protection in the United States, which was unprecedented in terms of the scale of rallies and mass participation, as well as the improvement in citizens' ecological awareness and the impact on the world's environmental history. This movement greatly brought into play the power of citizens' extensive participation in ecology, triggered the reform of citizens' ecological concept, and improved citizens' ecological consciousness. Obviously, this approach to cultivate citizens' ecological awareness is worth learning from [17]. At present, Chinese citizens have weak ecological awareness and a lack of ecological consciousness. Therefore, it is urgent to cultivate the ecological consciousness of Chinese citizens to take the initiative to undertake relevant environmental protection affairs. The government should play a leading role in overall planning, setting up specialized training institutions, and providing more economic support. The cultivation of Chinese citizens' ecological awareness is temporarily dependent on the guidance of the government. With the popularization of the cultivation of ecological awareness and the enhancement of citizens' awareness level, citizens will gradually develop conscious ecological awareness, and the era of national environmental protection is expected, relying on the nurturing power of community organizations. The high level of ecological consciousness of foreign citizens lies not only in the bottom-up ecological education mechanism and ecological practice, but also in the spontaneous leading and exemplary role of various nongovernmental organizations in society. Since the 1980s, community organizations in Western developed countries have played an increasingly significant role in the education of environmental protection and ecological civilization. The UK adopted self-government early on, allowing residents to be their own masters and take good care of the environment as if they were their own homes. This kind of autonomous community organization brings together a large number of people, integrates many educational functions, edifies and strengthens citizens' strong environmental awareness, and creates an atmosphere of ecological environmental protection in which all members participate and the whole people consciously. In contrast, Chinese community organizations are only in the initial stage, and under the administrative intervention of the government, they are not fully equipped with personnel, and carrying out ecological activities is just a government action with strong purpose and lack of consciousness and initiative. In the new era, community organizations can carry out multichannel and multiform environmental protection publicity and education activities under the administrative guidance of the government. Community organizations should constantly optimize the personnel structure and professional quality improve the ecological awareness, professional ability, and management level of community workers. Community is an important carrier of social management. As the most basic social grassroots organization, community can give full play to its social capital advantage in the process of direct communication with citizens, which plays an important role in further popularizing and enhancing the ecological awareness of Chinese citizens. Implement the educational means of co-governance of Germany and France. Singapore enjoys the reputation of “garden city,” on the one hand, due to the government's high attention to and management of environmental protection affairs, and on the other hand, due to citizens' deep awareness of environmental protection [18]. To cultivate citizens' ecological awareness in China, we should also learn from Singapore's successful experience and adopt the method of co-governance between Germany and France. Through the compulsory and binding nature of law, we should get rid of all kinds of nonstandard behaviors in the field of ecology, establish mechanisms and systems with legal effect, establish citizens' ecological legal consciousness, and gradually realize the scientific and legal cultivation of citizens' ecological consciousness. Meanwhile, by a variety of publicity and education, a good environment is created for the cultivation of ecological consciousness among citizens, making them gradually establish an idea of an ecological legal system, enhance their ecological personality and quality, make them role models of environmental protection and ecological behavior, and train and develop them in accordance with the socialist core value system.

The article "Research on Citizen Participation in Government Ecological Environment Governance Based on the Research Perspective of “Dual Carbon Target”" was published in 2022. Journal: J Environ Public Health.

### 3.2. Expanding Ecological Awareness Education

The original ecological concept of citizens is changed and the education level of citizens' ecological awareness is improved. At present, China's ecological awareness education level is still in its infancy. In the new stage, citizens' ecological awareness education needs to be improved in terms of educational content, methods, subjects, and objects. First, enrich the content of ecological awareness education. At present, the level of ecological awareness education in China is still in its primary stage, with small scale, imperfect system, low influence, and low education level. In the new stage, the education of citizen ecological consciousness needs to be improved in the aspects of education content, mode, subject, and object. First, enrich the content of ecological awareness education. At present, the main content of ecological awareness education in China is the popularization and education of popular science knowledge about ecological environment, which helps to provide basic knowledge for the cultivation of ecological awareness of citizens and improve their ecological awareness level. In the new era, citizens' ecological awareness education should constantly integrate new contents and strengthen the education of citizens' ecological national conditions, ecological legal system, ecological tourism, ecological consumption, and other contents [19]. The education of ecological national conditions is to publicize and educate citizens about the current situation and problems of China's ecological environment. Ecological legal education is to enable citizens to understand the relevant laws and regulations of ecological environmental protection. Ecological consumption education is to advocate the concept of green consumption, pay attention to the harmony between man and nature, and save resources and consume scientifically while pursuing a comfortable life. Ecotourism education is to instill ecotourism knowledge to tourists, guide tourists' ecological values and behavior patterns with a definite aim, reduce their unnecessary personal needs and consumption, awaken tourists' strong ecological consciousness, and make tourists become rational and full of feelings of ecotourism. Second, the way of ecological awareness education is improved. At present, the main methods of ecological awareness education in China include school curriculum education, media publicity, and personnel training. In the new period, we should innovate the way of ecological consciousness education and realize the organic combination of explicit education and implicit education. Explicit education is to inculcate and publicize the content of ecological education to the educators through collective teaching, training, and thematic discussion activities through open propaganda and educational means, so as to improve their ecological awareness. Implicit education is to integrate good ecological consciousness into specific behaviors and habits of daily life in the way of spring breeze and rain, or a scene or a story, and consciously practice the concept of ecological protection. Being civilized, loving the environment, and consuming less can make citizens truly understand the importance of the ecological environment to human existence and realize harmony between man and nature. It is an effective way to strengthen the ecological consciousness of Chinese citizens to combine the explicit theme education with the hidden life infiltration and make the education of civic ecological consciousness constantly perfect in practice. Third, the subject and object of ecological consciousness education is expanded. At present, the main body of ecological awareness education in China is relatively single, which is mainly undertaken by schools. To this end, all resources and forces, including government, enterprises, nongovernmental organizations, and mass media, should be mobilized through multiple channels and at multiple levels. Here, the government can play a leading role to ensure the smooth development of educational activities; mass media can play the role of information platform to expand the popularization of ecological education; enterprises can realize green production and circular economy mode by improving employees' ecological literacy; and nongovernmental organizations should be good at communication to implement educational activities. At the same time, the object of ecological awareness education should be continuously expanded [20]. In school education, the whole process of education from kindergarten to university is realized, and everyone at every stage experiences ecological awareness education.

The article "Research on Citizen Participation in Government Ecological Environment Governance Based on the Research Perspective of “Dual Carbon Target”" was published in 2022. Journal: J Environ Public Health.

### 3.3. Strengthening Government Guidance

Positive guidance is to strengthen the government to foster citizen participation in the ecological practice ability that can improve the level of citizens' ecological consciousness education to a certain extent, the citizens' ecological consciousness change and enhanced; however, citizens' ecological consciousness shape cannot just stay on theory education level; it is a practical problem, be badly in need of citizens in the practice of the ecological environment governance in China, local ecological cultivation. In the new era, the government should strengthen the positive guidance and cultivation of citizens in order to improve citizens' ecological awareness from the perspective of ecological and environmental collaborative governance. One is to enhance citizens' awareness of participating in ecological practice. As an agricultural country with a history of thousands of years, influenced by traditional economic, political, and culture, the citizen' ecological knowledge is still very scarce, the ecological idea is narrow, the ecological environment in collaborative governance problems often exist, and passive and obedient negative mentality leads some citizens to participate in the process of ecological practice which often show that it cannot participate in or displacement of mind. This has greatly hindered citizens' ecological practices and affected ecological environmental governance activities.

Strengthening the status and participation of nonprofit organizations and grassroots institutions and guiding citizens to actively participate. Debate mechanisms and dialogue mechanisms for civil participation can be appropriately set up to strengthen communication between government departments and citizens. The Internet can be used to encourage nonprofit NGOs to open corresponding public opinion polling forums, and the government can also open forum channels through official channels. The interests and groups represented by each organization are different. Through the forums of each organization, citizens can find the decision-making topics they are interested in and conduct public opinion surveys and statistics based on the status of the interest groups represented by each organization. This approach simplifies the classification process after the government collects information, improves the efficiency of information collation, enables citizens to obtain corresponding feedback faster, and promotes citizen participation; government departments can also further understand where citizens stand and from which aspects After consideration, corresponding administrative demands will be put forward. In this way, the government can consider the environmental background of citizens and propose better solutions or appeasement when dealing with slightly conflicting opinions.

The article "Research on Citizen Participation in Government Ecological Environment Governance Based on the Research Perspective of “Dual Carbon Target”" was published in 2022. Journal: J Environ Public Health.

### 3.4. Improve the Legal System and Enhance the Rule of Law

Deng Xiaoping once pointed out that in order to protect the people's democracy, the rule of law must be strengthened, and democracy must be institutionalized and legalized, so that the system and laws will not change due to changes in leaders, nor changes in leaders' views and attention. The report of the 19^th^ National Congress of the Communist Party of China also clearly pointed out that: we must adhere to the organic unity of the party's leadership, the people as masters of the country, and the rule of law; expand the people's orderly political participation; and ensure that the people implement democratic elections, democratic consultations, democratic decision-making, democratic management, and democratic governance in accordance with the law, supervision. Therefore, in order to promote civic participation, it is necessary to create a participatory democratic political and cultural atmosphere, encourage the public to establish a sense of participation, cultivate a participatory legal culture, enhance civic confidence in participation, establish a sense of participation, and transform civic participation from passive participation to active participation. A service-oriented government is a government ruled by law. At this stage, due to imperfect laws and regulations and the lack of specific implementation measures for participation in procedures, it is difficult to mobilize the enthusiasm and initiative of some local citizens to participate. To solve this problem, we must establish and improve the laws and regulations related to citizen participation, improve the democratic degree of citizen participation, and promote citizen participation.

First of all, promote citizens' participation in legislation, realize participation in the rule of law, and use special laws to protect citizens' right to participate in administrative decision-making. A complete set of legal protection system should be established for citizens' participation in administrative decision-making. From the legal perspective, citizens' participation in government management is a citizen's right, and the right of citizens to participate in administrative decision-making should be guaranteed by law. As the current stage of my country's citizens as the subject of participation has not been clarified at the legal level, the participation of citizens in public decision-making cannot be relied upon. Therefore, relevant laws should be promulgated as soon as possible to make citizens' participation in administrative decision-making legal, and the policy scope of citizens' participation in administrative decision-making should be clearly defined in law; the government and citizens' behavior should be regulated procedurally; and the forms, channels, and steps of participation should be regulated, making procedural specifications. In addition, it is necessary to clearly stipulate the remedies and solutions after the citizens' right to participate in the administration is violated and to hold accountable for the violations of citizens' right to participate in administrative affairs. Second, local governments should be appropriately encouraged to issue corresponding participation measures and regulations. In 2007, the Guangzhou Municipal Government issued my country's first standardized local management method for citizen participation in administrative legislation, “Guangzhou Municipal Regulations and Public Participation Measures.” Therefore, it is necessary to establish more convenient participation methods according to local conditions and in accordance with the needs of local people. Among them, the participation process must be clearly defined, the decision-making process must be made public, a feedback system must be established, and public supervision must be accepted. For the relevant regulations and regulations extended by the Participation Law, it is necessary to make clear and feasible provisions for the participation process in combination with the actual local conditions and clarify which decision-related matters need to be determined from the three stages before, during, and after policy formulation. Citizen participation, through which channels, how to understand the content of decision-making, and how to respond to citizens' suggestions and opinions are very important. A sound legal guarantee system can ensure that citizens' participation has laws to abide by, laws must be followed, violations must be punished, citizens' rights are guaranteed, participation events are dealt with in a standardized way, and the sustainable and sound development of citizen participation is promoted.

The article "Research on Citizen Participation in Government Ecological Environment Governance Based on the Research Perspective of “Dual Carbon Target”" was published in 2022. Journal: J Environ Public Health.

## 4. Conclusion

With the growth of people's demand for a better life, the public's demand for the rural ecological environment is also increasing. At present, the environment of many rural areas is deteriorating and the sewage is flowing, posing a major challenge to the governance of the rural ecological environment. Therefore, improving the ability and level of rural ecological management is the key to winning the tough battle of rural ecological management, and citizen participation in rural ecological management is more important for improving the ability and level of rural ecological management. Therefore, this article aims at the problems that the relevant legal systems in the current ecological governance are not perfect, the awareness of citizens' participation is weak, and the methods of citizen participation are difficult to determine, which seriously hinder the participation of citizens, to improve citizens' awareness and ability to participate in ecological environment governance to improve the citizen participation mechanism in my country's rural ecological environment governance.

## Figures and Tables

**Figure 1:** Comparison of public ecological environment behavior in China.

**Figure 2:** Citizens' attention to environmental events.

**Figure 3:** Degree of citizens' understanding of ecological governance.

**Figure 4:** Access to information for citizens.

**Figure 5:** Interviewees in different units pay attention to ecological environment information.

**Figure 6:** Different interviewees focus on ecological and environmental governance.

**Figure 7:** Enthusiasm for citizen participation.

**Figure 8:** Changes of harmless treatment capacity.

**Table 1:** Public participation intention and participation method.

Participation comments	Proportion (%)	Participation method	Proportion (%)
Very willing	47.5	Promote environmental knowledge	11.59
More willing	36.82	Participate in the public welfare activities of the government and social organizations	34.32
Reluctance	12.5	Start from the smallest things around you to protect the environment	51.36
Does not matter	3.18	Suggestions for pollution control rules and regulations	2.73

## Data Availability

The dataset used to support the findings of this study is available from the corresponding author upon request.
